The article "Influence of Healthy Physical Fitness on the Teaching of Aerobics Course Based on Big Data Mining Technology" was retracted in 2023. Reasons: signs of a paper mill; suspected computer-generated content; unreliable results or conclusions; lack of ethics approval or compliance.

# Influence of Healthy Physical Fitness on the Teaching of Aerobics Course Based on Big Data Mining Technology

**DOI:** 10.1155/2021/9755214

**Published:** 2021-12-22

**Authors:** Laipeng Xiao

**Affiliations:** Tianjin University of Sport, Tianjin, China

## Abstract

Healthy physical fitness is one of the hot topics discussed by scholars at home and abroad in recent years, and it is a key indicator for evaluating students' physical function and body shape. Aerobics, also known as bodybuilding, means that the body and health of students should have a better promotion effect, but in reality, many students found that after elective aerobics, body shape and health level basically did not improve, which is related to the setting of aerobics courses, especially the lack of physical training. Aerobics and other sports have common requirements in physical training, such as strength quality, speed quality, endurance quality, agility quality, and flexibility quality. This article is aimed at studying the impact of healthy physical fitness based on big data mining technology on the teaching of aerobics. On the basis of analyzing the process of data mining, the composition of healthy physical fitness, and the role of aerobics, it is used to test students in a certain university through experimental methods and statistical methods. Carry out aerobics teaching experiment, and compare and analyze the data measured by the experimental samples. The experimental results show that the use of healthy physical fitness in aerobics teaching can effectively promote the learning and improvement of aerobics skills.

## 1. Introduction

The 21st century is a new era of vigorous development of higher education. In the context of the market economy era, cultivating talents with high competitiveness, innovative and entrepreneurial spirit, and integrated development of multiple comprehensive qualities is one of the important goals and directions of the priority development of colleges and universities [1, 2]. Sports teaching has always been a major part of higher education. A good body of students is very important to students' research and life. For this reason, there is an urgent need to improve and establish a sports research system that matches the educational development policy and the national development strategy [3, 4].

When the aerobics athletes and other sports athletes can be of the same body level, which is conducive to the development of aerobics, competitive aerobics and other aerobics are different, aerobics movement difficulty and team changes have the same place, and they can be said to be closely related. Because of abundant practice and theory research, aerobics develops rapidly and has relatively complete practice and theory foundation. Through consulting relevant information, we find that there are relatively few studies on calisthenics physical training.

The article "Influence of Healthy Physical Fitness on the Teaching of Aerobics Course Based on Big Data Mining Technology" was retracted in 2023. Reasons: signs of a paper mill; suspected computer-generated content; unreliable results or conclusions; lack of ethics approval or compliance.

After sorting out the literature, it is found that there is less research on the teaching of aerobics for healthy physical fitness. Some scholars believe that when teaching students healthy physical fitness. First of all, teachers should clarify their knowledge of physical fitness theory and express the deep meaning of physical fitness theory to students. There are specific reasons for choosing the content of healthy physical fitness. Through teaching, the teaching experience will be accumulated, and the teaching experience will be gradually enriched after the accumulation of time. Therefore, the physical health of the students is improved [5, 6]. Some scholars mainly discuss the influence of aerobics on education when studying the teaching methods of healthy physical fitness. The scholar took 180 students as the survey object. The experimental results show that the health and physical fitness indicators of the experimental group students have been strengthened. It shows that healthy physical training has a great role in improving the physical condition of students [7, 8]. Some researchers start with enriching the content of physical education in our country. Let aerobics teaching no longer be boring and innovative teaching methods. At the same time, improve the physical condition of students. Therefore, a healthy physical fitness aerobics teaching is designed [9, 10]. There are also researchers who experiment with middle school students, who always take “health first” as their guiding ideology [11, 12]. Combining the above research results, it is hoped that through the research of this article, a novel teaching method can be explored and the current teaching situation can be changed. At the same time, it provides training methods for the healthy development of students.

This paper is based on consulting a large number of topics about “health fitness” and “aerobics courses,” combining the process of data mining, the composition of health fitness, and the role of aerobics, using experimental and statistical methods to treat the students of a certain university. Aerobic exercise teaching experiments were performed, and data measured from experimental samples were compared and analyzed.

## 2. Research on the Influence of Healthy Physical Fitness on the Teaching of Aerobics Course Based on Big Data Mining Technology

### 2.1. The Process of Data Mining

#### 2.1.1. Determine the Analysis Object

Determining what to analyze is the most important step in the entire data mining process. Before data mining, you need to determine the purpose of data mining analysis, such as the purpose of the experiment and the problem to be solved. Only by understanding and learning the knowledge of related industries in advance can we more effectively find valuable data information according to our needs. If you do not know the purpose of the research, it is difficult to achieve people's expectations and results [13].

The article "Influence of Healthy Physical Fitness on the Teaching of Aerobics Course Based on Big Data Mining Technology" was retracted in 2023. Reasons: signs of a paper mill; suspected computer-generated content; unreliable results or conclusions; lack of ethics approval or compliance.

#### 2.1.2. Data Preprocessing

*(1) Select Data*. Once the purpose and purpose of the analysis are determined, the data needs to be analyzed to understand which data can support the business and which data can be used to solve the problem. The goal of this stage is to select the appropriate data set, determine the most relevant data set to the object, and lay a solid foundation for a future work [14].

*(2) Data Cleaning*. After verifying the data set, the data needs to be preprocessed. At this stage, it may be found that there are missing data, duplicate values, outliers, etc. The missing value generally depends on the degree of the missing value. If the missing part is small, you can use the average to fill it; if the missing value is large, delete the attribute or this data immediately [15].

*(3) Data Transformation*. After completing the above steps, you need to convert the data to another format. Common methods include standardized or standardized data. A wise data conversion model can greatly improve the efficiency of data mining.

*(4) Feature Engineering*. Feature engineering defines the entire model online. This can be divided into artificial features and mechanical features. Artificial features start from a practical point of view and create features based on experience, so you need to have an in-depth understanding of your business. Machine functions refer to functions directly created by algorithms such as PCA, neural networks, and other methods.

#### 2.1.3. Data Mining

Data mining is the process of analyzing and processing the received data set. Feature engineering determines the upper limit of the entire model, so the choice of model and parameters is to approach this upper limit infinitely. In the process of building the model, the most suitable algorithm needs to be selected. Available algorithms include machine learning algorithms and deep learning algorithms. Available algorithms include ranking, regression, cluster analysis, and correlation analysis. Second, choosing the most appropriate analysis model before completing the project can significantly improve the efficiency of the mining facility.

#### 2.1.4. Overall Analysis

Once the results of the excavation investigation are obtained, a systematic assessment should be carried out at all stages of the entire excavation process. Remove irrelevant information or redundancy in the mining results. If the mining results significantly deviate from expectations, it may be necessary to review all the previous steps and may change a new analysis model or mining algorithm. Therefore, global analysis is a model optimization process that always exists and runs multiple times.

The article "Influence of Healthy Physical Fitness on the Teaching of Aerobics Course Based on Big Data Mining Technology" was retracted in 2023. Reasons: signs of a paper mill; suspected computer-generated content; unreliable results or conclusions; lack of ethics approval or compliance.

### 2.2. The Composition of Healthy Physical Fitness

#### 2.2.1. Cardiorespiratory Endurance Fitness

Cardiopulmonary endurance, also known as aerobic endurance, refers to the aerobic capacity of the human body during long-term exercise of large muscle groups. The level of cardiopulmonary endurance is mostly related to the normal functions of the cardiovascular system and the human respiratory system. The level of cardiorespiratory endurance is mainly determined by the body's ability to receive and transport oxygen, and the body's ability to use air. Cardiorespiratory endurance levels are closely related to human health. Good human body should have long-term effective work ability, to ensure that the body can quickly reduce the fatigue after work, so as to effectively restore the function, and good heart and lung endurance is inseparable.

#### 2.2.2. Muscle Fitness

Muscle health is one of the key technologies for human beings to cope with the difficulties in life. It can include energy and endurance. The first refers to the force with which the muscle overcomes the greatest obstacle when it is tightened or compressed, and the second refers to the development of the muscle under a specific load. As the duration of the work increases, maintain the strength of the contraction or the maximum number of repetitions. The necessary energy and endurance are essential for daily activities, work environment, and fitness. However, once the intensity is not suitable for work, it will cause local muscle contraction, bone degradation, and physical weakness and threaten life in the most serious cases.

#### 2.2.3. Body Composition

The sum of the weight of adipose tissue and the weight of nonfat tissue is called the overall weight. Nonfatty tissues include bone, muscle, and water. Lean body mass is also called the nonfat body mass of the body. Therefore, the proportion of body fat tissue proportion and lean body mass in total weight represents the body composition of the human body. Because fat has important physiological functions such as generating heat, maintaining body temperature, storing energy, and protecting the body, increasing the fat concentration in the body composition will inevitably reduce the body's muscle composition, thereby reducing the basic level of physical activity and metabolism.

The article "Influence of Healthy Physical Fitness on the Teaching of Aerobics Course Based on Big Data Mining Technology" was retracted in 2023. Reasons: signs of a paper mill; suspected computer-generated content; unreliable results or conclusions; lack of ethics approval or compliance.

#### 2.2.4. Body Flexibility and Fitness

Body flexibility refers to the range of joint movement. This is within the allowable range for bending and stretching of the muscles, tendons, and ligaments around the joints. In the maximum movement area of the limbs, various movements can be completed flexibly and at the same time prevent damage to the joint muscles and joints. Reducing the range of motion of a joint will limit the range of motion of a particular joint. Without preparation, muscle tension, pain, bruises, fractures, and other problems may occur in local tissues of the body, which will damage the health of the body.

### 2.3. The Role of Aerobics

1. The positive effects of aerobics in promoting the development of campus culture. Aerobics is not just a sport that is welcomed by the majority of students and is of general interest. At the same time, it drives the development of the entire campus culture and integrates with it and develops in harmony. The new type of sports integrated with art functions is also the main component and expression of the entire campus culture and, to a considerable extent, contains the sports culture, entertainment culture, art culture, and psychological culture of the entire campus culture. It is also used in the construction of campus culture
2. The role of aerobics in national fitness. During the “Twelfth Five-Year Plan” for sports development, aerobics has a unique advantage in the country's physical fitness. It is simple, easy to use, and highly flexible and has low investment and has a wide range of categories for the crowd. It creates a fashion trend pioneer for bodybuilding and perfect body shape, effectively improving human body functions and promoting healthy growth of the human body. Aerobics is a national fitness hotspot, an important link between teaching and lifelong sports in physical education schools, and the cornerstone of the nation's national health plan
3. The role of aerobics in teaching is to make many students have the courage to express their own psychology and, at the same time, allow them to make physical adjustments in a happy learning environment, so that many students begin to have the awareness of exercise, and the habit of exercise has gradually begun to form. Aerobics has created an atmosphere of active exercise and healthy life in junior high school campuses and cultivated a lifelong awareness of sports. Aerobics training is one of the key teaching contents of physical education elective courses in colleges and universities. Students' physique is particularly good, which can also relieve students' fatigue and vitality after experiencing a stressful study and life. In this way, students develop the good habit of conscious exercise, cultivate the overall aesthetic level, strengthen the friendship and exchanges between alumni, and enrich the campus culture
4. The influence of aerobics on mental health can not only improve the physical condition but also change the mental environment, promote physical and mental health, and prevent and treat mental illness; aerobics exercise can activate students' learning motivation, adjust emotions, and expressiveness. And it can also enhance students' academic performance and mental stability. It also has a positive impact on students' psychological nursing and psychological teaching. It can not only improve interpersonal relationships, relieve the pressure of scientific research, and stimulate students' pursuit of beauty and yearning for beauty but also improve psychological quality and increase artistic appreciation; mass aerobics has a great impact on mental health. Through mass aerobics exercises, it enables participants to adjust mood, enhance self-confidence, stabilize emotions, adapt to environmental changes, expand the range of making friends, cultivate and improve social skills, and maintain a wide range of interests, enjoy life, etc., thereby improving individual mental health and satisfaction

The article "Influence of Healthy Physical Fitness on the Teaching of Aerobics Course Based on Big Data Mining Technology" was retracted in 2023. Reasons: signs of a paper mill; suspected computer-generated content; unreliable results or conclusions; lack of ethics approval or compliance.

## 3. Experiment

### 3.1. Research Objects

This article takes the 2020 students of a university in this province as the research object and randomly selects two aerobics selection classes. Class A is the experimental class (47 students), and Class B is the control class (47 students), with a total of 94 students. All of the students come from different departments and majors. They had a relevant knowledge of their basic situation before the experiment. Subjects did not often participate in physical exercise, but their physical health, cardiopulmonary function, and other aspects were normal.

### 3.2. Research Methods

#### 3.2.1. Experimental Method

Combine healthy physical fitness with aerobics for experimental analysis. Through the experimental group aerobic exercise intervention, the subject health and fitness measures were tested following the prescribed exercise measurement and evaluation rules, and the test data results were compared to the control group. To compare, explore the effect of healthy physical fitness intervention in aerobics class on the healthy physical fitness of college students.

#### 3.2.2. Data Statistics Method

The statistical analysis of the health fitness index of 94 college students before and after the aerobics exercise cycle was carried out, and the results were expressed in terms of mean ± standard deviation (*M* ± SD). Using sPSS14.0 statistical software, paired *T* test and independent sample *T* were performed. In detection, when *P* > 0.05, it means that there is no obvious change, *P* < 0.05 means that there is a certain change, and *P* < 0.01 means that the change is very obvious. The *T* test calculation formula is as follows:

(1) $$\begin{array}{c} t=\bar{X}-\mu /\left(\sigma_{X}/\sqrt{n-1}\right). \end{array}$$

If the sample is a large sample (*n* > 30), it can also be written as

(2) $$\begin{array}{c} t=\bar{X}-\mu /\left(\sigma_{X}/\sqrt{n}\right). \end{array}$$

Here, *t* is the deviation statistic between the sample mean and the overall mean, and *n* is the sample size.

The article "Influence of Healthy Physical Fitness on the Teaching of Aerobics Course Based on Big Data Mining Technology" was retracted in 2023. Reasons: signs of a paper mill; suspected computer-generated content; unreliable results or conclusions; lack of ethics approval or compliance.

## 4. Discussion

### 4.1. Test Comparison of Physical Fitness Index

Before starting the teaching experiment in a university, this article tested and collected the basic information of the experimental group and the control group and confirmed the difference test of the experimental group and the control group's health and physical conditions. The situation is shown in Table 1 and Figure 1. Before the experimental intervention, the physical status of the students in the experimental group and the control group was basically at the same level. The index data of the heart rate, vital capacity index, seated forward bending, and forearm grip strength of the step experiment were not much different, and there was no significant difference.

The data of the experimental class and the control group after the experiment is shown in Table 2 and Figure 2. It can be found that the performance of the students in the experimental class is comparable in the three indicators of cardiopulmonary endurance, muscle strength, and flexibility, and the test results are significantly different. Increasing the content of healthy physical education activities in the university elective aerobic sports courses and strengthening the practice of various targeted skills can effectively improve students' physical quality.

It can be seen from Table 2 and Figure 2 that after the experiment, the average level of the experimental class in vital capacity, flexion, forearm grip, and sit-ups was significantly higher than that of the control class students. After the test (*P* < 0.05), the experimental class and there are significant differences in these four physical fitness indicators for students in the control class.

### 4.2. Comparison of Aerobics Performance

In order to verify the effect of healthy physical fitness on aerobics teaching, this article compares the test results of aerobics between the experimental class and the control class.

Through the results of the teaching experiment combining healthy physical fitness in the aerobics class, it can be seen from Table 3 and Figure 3 that after the experiment, the maximum aerobics performance of the students in the experimental class is 85 points, the minimum is 53 points, and the average is 72.98 points; the maximum aerobics performance of the students in the control class is 81 points, the minimum is 51 points, and the average is 68.24 points. According to the data, the aerobics performances of the students in the experimental class are all higher than the aerobics performance of the students in the control class by 4.74 points and have a very significant difference (*P* < 0.01). This shows that the use of healthy physical fitness in aerobics teaching is effective. To a certain extent, healthy physical fitness can promote students to learn and master aerobics skills.

The article "Influence of Healthy Physical Fitness on the Teaching of Aerobics Course Based on Big Data Mining Technology" was retracted in 2023. Reasons: signs of a paper mill; suspected computer-generated content; unreliable results or conclusions; lack of ethics approval or compliance.

A further comparative analysis of male and female students was made through the results of the teaching experiment combining healthy physical fitness in the aerobics class. The results from Table 4 and Figure 4 show that the average score of the male aerobics skill test in the experimental course after the experiment is 69.96, which is higher than that of the control class, and has a very significant difference (*P* < 0.01); after the experiment, the average value of the girls' aerobics performance in the experimental class is 76.76, which is 5.22 points higher than that in the control class, with a significant difference (*P* < 0.05). This shows that the use of healthy physical fitness in aerobics courses can more effectively promote the mastery and improvement of aerobics techniques.

## 5. Conclusions

From the theory of teaching and education optimization, modern educational technology has a close relationship with college aerobics teaching. Through the theory, we can optimize the education mode and upgrade the education technology, so as to maximize the advantages of teaching effect. Creating good material conditions to ensure teaching, improving teachers' updating of education methods, and optimizing education contents are the basis of improving education quality. Therefore, good teaching mode, efficient teaching tools, and means for the development of efficient aerobics have played a key role. In the field of aerobics teaching, the application of modern educational technology to assist aerobics teaching is a powerful embodiment of teaching and teaching optimization theory in teaching methods and teaching conditions.

This article introduces healthy physical fitness into aerobics courses to carry out practical exploration, which can not only improve students' understanding of healthy physical fitness but also realize the improvement of students' aerobics skills while improving their health and physical fitness levels, so that students can develop aerobics as an exercise. Lifelong physical exercise programs improve the health of students and continue to decline. Students respond to the needs of colleges and universities to improve their own health and physical fitness.

The article "Influence of Healthy Physical Fitness on the Teaching of Aerobics Course Based on Big Data Mining Technology" was retracted in 2023. Reasons: signs of a paper mill; suspected computer-generated content; unreliable results or conclusions; lack of ethics approval or compliance.

## Figures and Tables

**Figure 1:** Comparative analysis of test results of students' health and physical fitness index before experiment.

**Figure 2:** Comparative analysis of test results of students' health and physical fitness index after experiment.

**Figure 3:** Comparison of the results of aerobics skills test between the experimental class and the control class.

**Figure 4:** Comparison of the results of aerobics skills test between male and female students in the experimental class and the control class.

**Table 1:** Comparative analysis of test results of students' health and physical fitness index before experiment.

Test items	Experimental class	Control class	*t*	*p*
Step experiment	119 ± 10.36	118.27 ± 11.14	3.45	>0.05
Vital capacity	3093.48 ± 824.32	3041.25 ± 812.65	4.997	>0.05
Sitting forward bending	18.54 ± 7.62	18.63 ± 6.12	1.324	>0.05
Forearm grip	26.524 ± 2.641	26.438 ± 2.84	0.33	>0.05
Sit-ups	27.64 ± 5.147	27.851 ± 4.657	1.533	>0.05

**Table 2:** Comparative analysis of test results of students' health and physical fitness index after experiment.

Test items	Experimental class	Control class	*t*	*p*
Step experiment	113 ± 9.21	118.27 ± 11.14	3.483	<0.05
Vital capacity	3524.26 ± 841.74	3041.25 ± 812.65	4.322	<0.05
Sitting forward bending	25.45 ± 5.33	19.65 ± 4.82	1.324	<0.05
Forearm grip	29.47 ± 2.35	26.43 ± 2.86	7.367	<0.05
Sit-ups	33.54 ± 5.751	27.42 ± 46.812	6.274	<0.05

**Table 3:** Comparison of the results of aerobics skills test between the experimental class and the control class.

Test subject	Maximum value	Minimum value	Average value	*t*	*p*
Experimental class	85	53	72.98	-5.08	<0.01
Control class	81	51	68.24		

**Table 4:** Comparison of the results of aerobics skills test between male and female students in the experimental class and the control class.

Test subject	Gender	Maximum value	Minimum value	Average value	*t*	*p*
Experimental class	Male	79	53	69.96	4.58	<0.01
Control class	Male	79	51	65.84		
Experimental class	Female	85	56	76.76	3.02	<0.05
Control class	Female	81	55	71.54		

## Data Availability

The data underlying the results presented in the study are available within the manuscript.
